# A Novel Approach to Skin Lesion Segmentation: Multipath Fusion Model with Fusion Loss

**DOI:** 10.1155/2022/2157322

**Published:** 2022-07-29

**Authors:** Adi Alhudhaif, Hakan Ocal, Necaattin Barisci, İsmail Atacak, Majid Nour, Kemal Polat

**Affiliations:** ^1^Department of Computer Science, College of Computer Engineering and Sciences in Al-kharj, Prince Sattam bin Abdulaziz University, Saudi Arabia; ^2^Computer Engineering (FT), Gazi University, Emniyet Mh., Milas Sk. No: 30, 06560 Yenimahalle, Ankara, Turkey; ^3^Gazi University, Technology Faculty, Computer Engineering, Ankara, Turkey; ^4^Department of Electrical and Computer Engineering, Faculty of Engineering, King Abdulaziz University, Jeddah 21589, Saudi Arabia; ^5^Department of Electrical and Electronics Engineering, Bolu Abant Izzet Baysal University, Bolu, Turkey

## Abstract

Segmentation of skin lesions plays a very important role in the early detection of skin cancer. However, indistinguishability due to various artifacts such as hair and contrast between normal skin and lesioned skin is an important challenge for specialist dermatologists. Computer-aided diagnostic systems using deep convolutional neural networks are gaining importance in order to cope with difficulties. This study focuses on deep learning-based fusion networks and fusion loss functions. For the automatic segmentation of skin lesions, U-Net (U-Net + ResNet 2D) with 2D residual blocks and 2D volumetric convolutional neural networks were fused for the first time in this study. Also, a new fusion loss function is proposed by combining Dice Loss (DL) and Focal Tversky Loss (FTL) to make the proposed fused model more robust. Of the 2594 image dataset, 20% is reserved for test data and 80% for training data. In test data training, a Jaccard score of 0.837 and a dice score of 0.918 were obtained. The proposed model was also scored on the ISIC 2018 Task 1 test images, whose ground truths were not shared. The proposed model performed well and achieved a Jaccard index of 0.800 and a dice score of 0.880 in the ISIC 2018 Task 1 test set. In addition, it has been observed that the new fused loss function obtained by fusing Focal Tversky Loss and Dice Loss functions in the proposed model increases the robustness of the model in the tests. The proposed new loss function fusion model has outstripped the cutting-edge approaches in the literature.

## 1. Introduction

Skin cancer is the 19th most commonly occurring cancer in men and women. There were nearly 300,000 new cases in 2018. Australia and New Zealand share the first two places in skin cancer patients [1]. In 2012, the total number of nonmelanoma skin cancer in the US population was estimated at 5,434,193. The total number of people treated for nonmelanoma skin cancer in the United States was estimated at 3,315,554 [2]. In the United States, $8.1 billion was spent for melanoma and nonmelanoma skin lesions, with a total cost of $4.8 billion and $3.3 billion, respectively [3]. Between 1994 and 2014, the number of nonmelanoma skin lesions reached 77% in the USA [4]. Approximately 90% of nonmelanoma skin cancers of nonmelanoma are associated with ultraviolet (UV) radiation from the sun [5]. The imaging technique used for the precise and efficient diagnosis of skin lesions is called dermoscopy. Dermoscopy allows doctors to diagnose and treat cancerous skin lesions in more detail by examining benign and malignant tumors on the skin that cannot be distinguished through the eye in more fact. Dermoscopy is performed with a hand microscope called a dermatoscope, which allows us to see under the skin surface in detail using polarized light. Thanks to the ABCD criteria used in the dermoscopy method, superior performance is obtained than other imaging methods [6]. However, precise and rapid skin lesion segmentation remains challenging due to diversity of skin lesions and the low difference between normal and lesioned skin. In addition, many artifacts such as hair strands and blood vessels cause problems during the segmentation [7–19].

For this reason, automated medical image segmentation is essential for facilitating the lesion's pathological diagnosis, planning treatment, and monitoring the disease's progress [20]. Second, some structures have various scales and shapes, such as skin lesions in dermoscopic views, making it challenging to create a previous shape model [21]. Besides, in magnetic resonance imaging (MRI), the location and orientation of some structures in the context of a large image, such as the placenta and fetal brain, can vary greatly [20, 22, 23]. Compared with the manual segmentation method, convolutional neural networks (CNNs) in many different organ segmentations have started to gain higher performance [24].

According to Taghanaki et al. [25], they replaced the jump links with the select-join-transfer (SAT) module to increase the segmentation robustness of the U-Net based model.

Jha et al. [26] proposed a binary parallel U-NET architecture using two U-NETs together.

Abhishek et al. [27] proposed a deep semantic neural network to improve the segmentation performance of deep learning-based networks.

Arora et al. [28] proposed a U-Net-based deep learning model using group normalization [29, 30].

Gu et al. [31] tried to propose a more robust model with multiple connections between layers by modifying the U-Net architecture. They also tried to increase the robustness of the model by adding a channel awareness module.

Goyal et al. [32] proposed a community network combining R-CNN and DeeplabV3C for segmentation of skin lesions.

According to Jiang et al. [33], they proposed the CSARM-CNN model that includes both channel and spatial attention modules for the segmentation of skin lesions based on deep learning C.

Lei et al. [34] proposed a general contentious network (GAN). The proposed model is a modified version of the U-Net network consisting of double layers.

According to San et al. [35], they proposed a community network combining FCN and DPN networks.

Ocal et al. [36] proposed an architecture fusing the 3D and 2D volumetric CNN (V-Net) networks for the segmentation of prostate images.

Ocal et al. [37] proposed a model combining ResUnet 3D and ResUnet 2D to segment MR prostate scans based on deep learning. They also proposed a new loss function that dynamically calculates the loss according to the mini-batch size.

In this article, information about data preprocessing and data augmentation is given in Chapter 2. In addition, information about the performance metrics used for the proposed model is given. The analyses of the proposed model are examined in the third section. In the 4th chapter, the analyses of the fusion model are evaluated. In addition, the performance results obtained were analyzed in comparison with other studies in the literature. In Chapter 5, the evaluations made in Chapter 4 are discussed, and various suggestions are made. In the 6th chapter, the conclusions of the proposed deep learning architecture are shared.

## 2. Materials and Methods

### 2.1. Dataset

In this study, the dataset was used for training and testing of the fusion method [21, 38]. The dataset consists of 2594 training images. The dataset from different institutes and various dermatoscopy types belongs to other anatomical regions of the patients containing various diagnostic challenges in the dermoscopic lesion images.

### 2.2. Preparing the Dataset

Deep learning methods usually require large datasets to produce better performance results. Therefore, image augmentation methods have been applied to the dataset to increase the number of images. First, 2594 images in the dataset were divided into different training (2075) and test (519) sets. The training images were then increased by applying horizontal and vertical flips, random rotation, random distortion, elastic transformation, and border data augmentation with the scaling and cropping method. The purpose of boundary data augmentation is to enable the proposed model better to detect the lesions' edges better. With the data augmentation methods applied, 72000 test images were obtained. This number is 92594 for the test set in the ISIC 2018 Challenge. That is, two different training datasets were created. The training model was used for 80% training and 20% validation compared with other models. Training images were pre-processed to achieve reliable and robust results. Next, contrast stretching was applied to make the lesions more prominent in the image. Contrast stretching always used the partial-based linear function that increased linearly and monotonously. Then, the sharpening algorithm was applied to the obtained images (with = 10). Thanks to sharpening, we tried to deal with the difficulty of fuzzy edges in images. Since the images are of many different sizes, and the proposed model is uniform, we resized all images to 512 × 512 dimensions.  Figure 1 shows examples of pre-processed and enhanced images.

### 2.3. Fusion Architecture

V-Net2D and U-Net + Resnet2D, which are the most used CNN models in biomedical image segmentation, have been fused in the proposed Fusion model. Milletari et al. [39] proposed V-Net architecture for volumetric, fully convolutional image segmentation. The proposed V-Net2D model for the fusion model is shown in Figure 2. As can be seen from the image, V-Net and U-Net are very similar [40]. However, the feature map is represented by squares in the figure. Additionally, it can be seen (orange line) that Vnet borrowed U-Net to superimpose the attribute map in the compressed path to complete the lost information (orange line). What needs a particular explanation here is that V-Net and U-Net's most significant difference is that V-Net uses the short circuit connection of residual block at each stage (gray route). It is equivalent to promoting residual block in U-Net. The residual block is Vnet's most significant improvement.

Besides, only one convolution is performed in the first stage of Vnet and twice in the second stage. The first and second layers in the compressing and decompressing stages are different from Unet's structure, which has the same number of convolution operations at each stage. Besides, we replaced the convolutions in the U-Net with the residual blocks shown in Figure 3. In this way, we have obtained the U-Net + Resnet2D model shown in Figure 4, where we achieve better performance than U-Net. The proposed fusion segmentation model is shown in Figure 5.

#### 2.3.1. The Encoder Stage

In each model, Xavier was employed for weight initialization and ReLU was employed as activation function [41]. In addition, ADAM was used for the optimization of the model [42]. In the V-Net2D model, the convolution layer in each channel consists of 3 × 3 filters. In addition, GN was used on the channels to normalize the feature maps. Unlike BN, GN normalizes groups of channels and calculates mean and variance for group normalization for each layer by performing both layer normalization (LN) and sample normalization (IN) simultaneously [7]. Unlike V-Net2D, U-Net + Resnet2D used BN instead of GN. In U-Net + Resnet2D, 2 × 2 maximum pooling was used, which halved the properties of the layer in the first four convolution blocks. Figures 2 and 4 show the encoder (left part of the image) preprocessed 512 × 512 × 1 input image fed into the first block. Also, the convolution layers increased 2× from 32 to 512 per block.

#### 2.3.2. The Decoder Stage

Low-resolution feature maps from the encoder are fed into the decoder section, upsampling images. As shown in Figures 2 and 4, upsampling (right part of the image) performs deconvolution, which is upsampling of feature maps from the downsampling stage. Low-resolution images with high-value feature maps are resized to the input image by performing many convolutions and merging operations in the decoder stage. Each convolutional layer in the decoder consists of 3 × 3 filters. ReLU is used as the activation function in each decoder layer. The output of the penultimate layers is fed into the 1 × 1 convolutional layer, which has the sigmoid activation function.

### 2.4. Evaluation Metrics

The proposed fusion model was scored in ISIC 2018 Challenge and using the most used performance metrics in the literature. The first of these metrics is the membrane similarity coefficient (DICE), which is a measure of the similarity of actual and predicted outcomes and is shown in Eq. (1). The Jaccard index (Jaccard), defined in Eq. (2), is a metric that calculates the ratio of similarity and difference of data samples. Accuracy (ACC), shown in Eq. (3), represents the percentage of correct predictions on the dataset. Sensitivity (Sens), defined in Eq. (4), is a percentage of the proportion of samples in test images estimated as true positive (TP). Sensitivity can also be defined as Recall. The Specificity (Spec), shown in Eq. (5), gives the percentage of correctly predicted lesion-free areas in the dataset. While DICE shows high performance in training in class imbalances, it is not as successful in estimating the test set. The metric defined to meet this challenge is the Tversky index function shown in Eq. (6).

(1) $$\begin{array}{c} Dice=\frac{2*TP}{2*TP+FP+FN}, \end{array}$$

(2) $$\begin{array}{c} Jaccard=\frac{TP}{TP+FN+FP}, \end{array}$$

(3) $$\begin{array}{c} Acc=\frac{TN+TP}{TN+TP+FN+FP}, \end{array}$$

(4) $$\begin{array}{c} Sens=\frac{TP}{TP+FN}, \end{array}$$

(5) $$\begin{array}{c} Spec=\frac{TN}{TN+FP}, \end{array}$$

(6) $$\begin{array}{c} TverskyIndex=\frac{TP}{TP+\alpha FN+\beta FP}. \end{array}$$

### 2.5. Loss Functions

A fusion loss model is obtained in the proposed model by fusing Focal Tversky Loss (FTL) and Dice Loss (DL), the most widely used loss functions in the literature. The loss functions used in the proposed fusion model are explained below.

#### 2.5.1. Focal Tversky Loss (FTL)

Another drawback of Dice Loss is the difficulty in segmenting small ROIs as there is no significant change in the loss. In this model, we used Dice Loss and Focal Tversky loss function (FTL), which constitute the fusion loss function. FTL is calculated using the in Eq. (7) formula. FTL can be called the fused form of cross-entropy with dice. It combines the loss curve's nonlinearity and controls how the function behaves at different samples [8].

(7) $$\begin{array}{c} FTL={\left(1-TI\right)}^{\gamma }. \end{array}$$

It is crucial that *γ* is chosen correctly in Eq. (7). If *γ* > 1, the loss function will focus more on false positives, making a worse prediction and classification. If it happens with *γ* < 1, then the loss function will focus more easily on the examples, and the training of the model will be faster. If we select *γ* = 0, the model will be no different from Tversky Loss. After trying different values for *γ* for the proposed model, we got the best result with *γ* = 0.75. For this reason, we set the *γ* value as 0.75 in all our training stages. We defined TI hyperparameters as *α* = 0.7 and *β* = 0.3 to better convergence of the proposed model to FP. If *α* = *β* = 0.5, the Tversky index will resemble the Dice Coefficient.

#### 2.5.2. Dice Loss (DL)

In the proposed model, Dice Coefficient (DSC) in Eq. (1). is taken as a reference as another loss function. DSC is a ratio of similarity of samples in two different datasets. DSC value takes values between minimum 0 and maximum 1. If Dice = 1, these two different clusters were matching each other perfectly. Conversely, if DSC = 0, it means that these two sets are entirely different from each other. Dice Loss is found by the 1-DSC formula to maximize overlap.

## 3. Calculation

### 3.1. Application Details

The hardware equipment used to evaluate the proposed model's performance must have sufficient Cuda and ram to train the model. Intel NVIDIA GTX 1080TI (11 GB) graphics card was used in the training of the proposed model. To calculate the final loss value of both models, the learning rate was set as 1*e* − 3 and the lot size = 4. The training of the models was carried out for 100,000 epoch. The models consisted of the proposed fusion model were trained separately on the preprocessed dataset. The tests were performed, as seen from the validation accuracy and loss values in Figures 6 and 7.

As shown in Figure 8, the small connected components were extracted from the test results obtained in the architectures forming the fusion model, using the SimpleITK.connected part in the Simple ITK model.

By comparing the prediction images obtained from the proposed model, the least related points are extracted. The final segmentation result was obtained by calculating the most overlapping regions.

### 3.2. Qualitative Analysis

The segmentation results and final segmentation result of each model in the proposed model are shown in Figure 5. In the figure, images obtained by the fusion of the two models with two different loss functions are demonstrated. Figures 6 and 7 show the graphical analysis of the models that form the proposed approach to validation accuracy and validation loss performed for 100,000 epochs.

### 3.3. Hardware Analysis

The recommended fusion model was tested using a NVIDIA Geforce GTX 1080 TI graphics card. The proposed model has been tested with other state-of-the-art models for the numerous model parameters, storage requirements, and extraction rates. There is no need for any operation that requires calculation before training in datasets. Training of each model took approximately from 4 to 6 hours with different loss functions. It took 15 minutes to calculate the overlap points of the V-Net and U-Net + Resnet2D models' results and find the final segmentation result.

## 4. Experimental Results

The proposed segmentation model's skin lesion performance was tested in the augmented ISIC 2018 dataset consisting of dermoscopic images. The proposed fusion model created by combining two different loss functions is thought to be a robust fusion model for lesion segmentation. One of the most important factors in this is the application of the border data augmentation method.

### 4.1. Comparison of the Proposed Model with Cutting-Edge Approaches

Table 1 shows the proposed framework's comparative study with other single methods using the ISIC 2018 dataset. The proposed fusion model is compared with the value in each loss function and fusion loss function of U-Net2D and V-Net2D. The augmented ISIC 2018 dataset achieved a Dice Coefficient of 0.92, surpassing the proposed architectural single models. This result was mainly achieved using Dice Loss and FTL as the fusion loss function best for small and complex lesion images. Besides, the proposed model has achieved better results compared to other single models.

Unlike other studies, the proposed model was also tested in the test dataset in the ISIC 2018 Challenge, and a dice score of 0.88 and a Jaccard score of 0.80 were obtained, as can be seen in Table 2. As can be seen from the table, the proposed model achieved from 2% to 4% more Jaccard scores than the single Vnet2D and Unet2D architectures thanks the new fusion loss function. The Dice and Sen performance results of the proposed model are consistent with the Jaccard score. The architecture based on the fusion model performed better than other single models in both the 20% test set and the ISIC 2018 Challenge test set and all segmentation processes.

Table 3 shows the proposed model's comparative results with other models on the ISIC 2018 dataset. Our fusion model obtained a dice score of 0.92 in tests on the 2018 Challenge dataset, surpassing the latest literature methods. Using attention gates (AG) and group normalization (GN), Attn_U-Net + GN achieved results closest to the proposed model. Although Attn_U-Net + GN performed well, the proposed model outperformed Attn_U-Net + GN in other performance metrics except for ACC. Another method that can be compared with the proposed model is SE_Unet. One of the reasons the proposed model outperforms other models is fusing the two best segmentation loss functions (DL + FTL) in the literature.

Figure 9 shows the visually estimated outputs of some complex samples in the ISIC 2018 1000 test set with the proposed approach and the models that make up the proposed model. As can be seen from the images, models with FTL gave better results. It is seen that V-Net2D models with FTL gave the closest results to the proposed approach.

The ground truth and predicted output of some complex samples in the 519 test images separated from the training dataset for training the proposed fusion model are shown in Figure 10.

## 5. Discussion

Maybe a little more training time will take as the recommended model is fusion. However, the testing phase will take almost the same time as the others. In a way, the study has been a comparative analysis study. We used BN in U-Net + Resnet2D and GN in V-Net2D. As can be seen from Tables 1 and 2, V-Net2D using GN gave more successful results. Besides, we had the opportunity to analyze Dice Loss and FTL comparatively in models with this study. FTL gave more successful outcomes than Dice Loss in the test results, as shown in Tables 1 and 2. Also, V-Net2D finished training 1.5 hours earlier than U-Net + Resnet2D. However, a more robust automatic segmentation model was obtained by fusing two different segmentation models and loss functions, most commonly used as backbones in the literature. Future studies can examine these two models and two different loss functions, and studies can be made on the new singular segmentation model and the loss function. However, there are still many challenging ways to achieve %100 flawless segmentation in all lesion imaging goals with AI studies used for diagnosis.

## 6. Conclusion

In this article, the proposed fusion model was created by fusing the two most robust networks, such as V-Net2D and U-Net + Resnet2D, which are the most used in the segmentation of skin lesions recently. Results have been trained and tested in the ISIC 2018 dataset. Images are entered into the proposed algorithm separately, containing gate vectors that separate essential information from lower-level information. GN in each CNN block in the upsampling and downsampling stage in the V-Net2D reduces the payload of precomputed statistics for images in groups. Also, a new loss function has been proposed by fusing the best loss functions DL and FTL. The novel fusion loss function proposed by combining DL and FTL has shown to be more suitable for skin lesion segmentation by obtaining higher performance metrics ratios in the experiments performed. The proposed fusion loss function can play a crucial role in challenging segmentation tasks. This created model has a highly desirable feature of outperforming existing essential segmentation networks. More tuning of the hyperparameters and adding more color space enhancements can provide better segmentation performances. Accuracy and Jaccard in the dataset were recorded as 0.95 and 0.84, exceeding the state-of-the-art segmentation techniques. The proposed model and fusion loss function are also tested in datasets from different medical fields to check their robustness and accuracy.

## Figures and Tables

**Figure 1:** Data augmentation of the training set. (a) 8 bit RGB image and (b) ground truth.

**Figure 2:** V-Net2d architecture.

**Figure 3:** Residual block.

**Figure 4:** U-Net + Resnet2d architecture.

**Figure 5:** Segmentation stages of the proposed model.

**Figure 6:** Unet+Resnet2D Validation Accuracy and Loss Results.

**Figure 7:** V-Net2D validation accuracy and loss results.

**Figure 8:** Removing small connected components. (a) U-Net + Resnet2D test result, (b) V-Net2D test result, and (c) U-Net-Resnet2D test result after removing the small connected pixels.

**Figure 9:** ISIC 2018 1000 test set prediction results. (a) Original image. (b) U-Net + Resnet2D + DL, (c) U-Net + Resnet2D+ FTL, (d) V-Net2D + DL, (e) V-Net2D + FTL, (f) proposed fusion model (DL: Dice Loss, FTL: Focal Tversky Loss).

**Figure 10:** Test results according to 519 splitted test set from the ISIC 2018 training set. (a) Input image, (b) image mask, and (c) predicted mask.

**Table 1:** Comparative analysis of proposed and the single methods (results of the 20% test set from the training set).

Method	Performance metrics				
	Dice	Jaccard	Acc	Sens	Spec
U-net + Resnet2D (with dice loss)	0.75	0.67	0.86	0.85	0.86
U-net + Resnet2D (with FTL)	0.87	0.79	0.88	0.87	0.88
V-Net2d (with dice loss)	0.88	0.81	0.91	0.90	0.91
V-Net2D (with FTL)	0.90	0.83	0.93	0.92	0.93
**Fusion model with fusion loss (ours)**	**0.92**	**0.84**	**0.95**	**0.95**	**0.96**

**Table 2:** Comparative analysis of proposed and the single methods (results of the ISIC 2018 test set).

Method	Performance metrics					
	T.Jaccard	Dice	Jaccard	Acc	Sens	Spec
U-net + Resnet2D (with dice loss)	0.56	0.72	0.64	0.86	0.85	0.86
U-net + Resnet2D (with FTL)	0.64	0.81	0.75	0.90	0.89	0.90
V-Net2d (with dice loss)	0.71	0.86	0.78	0.91	0.89	0.92
V-Net2D (with FTL)	0.72	0.87	0.79	0.91	0.92	0.91
**Fusion model with fusion loss (ours)**	**0.74**	**0.88**	**0.80**	**0.93**	**0.94**	**0.94**

**Table 3:** Comparative analysis of the proposed model with the cutting-edge methods in the literature.

Method	Performance metrics				
	Dice	Jaccard	Acc	Sens	Spec
Ensemble with CRF v3	0.90	0.84	0.95	0.93	0.95
SE_U-Net [28]	0.91	0.83	0.95	0.89	0.96
DAGAN [34]	0.89	0.83	0.93	0.95	0.91
DRU-Net [9]	0.86	0.76	—	0.88	0.92
Attn_U-Net + GN [28]	0.91	0.83	0.95	0.94	0.95
**Fusion model with fusion loss (ours)**	**0.92**	**0.84**	**0.95**	**0.95**	**0.96**

## Data Availability

Skin lesion analysis toward melanoma detection: A challenge at the 2017 international symposium on biomedical imaging (ISBI) hosted by the international skin imaging collaboration (ISIC). CoRR, abs/1710.05006. (https://arxiv.org/abs/1710.05006#). We have given the dataset from this database.
